RETRACTED

# Carbetocin Controls Intraoperative Blood Loss and Thickness of Myometrium in Scar Uterus Cases

**DOI:** 10.1155/2022/5477432

**Published:** 2022-10-04

**Authors:** Dongjing Sun

**Affiliations:** Department of Gynecology and Obstetrics, Hangzhou TCM Hospital Affiliated to Zhejiang Chinese Medicine University, Hangzhou, China

## Abstract

**Objective:**

To study the effect of carbetocin on intraoperative blood loss and thickness of myometrium during cesarean section with the scarred uterus at term pregnancy.

**Methods:**

Pregnant women with full-term gestational scar uterus who underwent cesarean section from March 1, 2021, to April 30, 2022, were retrospectively collected and divided into a reference group (using oxytocin) or a study group (using carbetocin). The clinical data of the two groups were retrospectively analyzed, and the operation time, intraoperative blood loss, hospital stay, uterine contraction effect, changes in the myometrium, and complications were compared between the two groups.

**Results:**

A total of 103 pregnant women were retrieved. There were 44 cases in the reference group and 59 cases in the study group. There were significant differences in operation time, intraoperative bleeding, hospital stay, postoperative adverse events, uterine fundus wall thickness, anterior wall thickness, posterior wall thickness, and uterine contraction effect between the two groups (*p*=0.0001, 0.005, 0.006, 0.001, 0.0004, 0.003, 0.001, and 0.005, respectively). There were no significant differences in estradiol (E2), luteinizing hormone (LH), or follicle-stimulating hormone (FSH) between the two groups before the surgery (*p*=0.596, 0.840, and 0.940, respectively), but there were significant differences after the surgery (*p*=0.011, 0.001, and 0.005, respectively).

**Conclusion:**

The use of carbetocin in the cesarean section of a full-term scar uterus is significantly effective in shortening the operation time, reducing the amount of intraoperative blood loss, and promoting the recovery of the uterus.

## 1. Introduction

The scar in the uterine wall area after cesarean section or myomectomy is defined as the uterine scar. A second cesarean section is generally performed after the scarred uterus is pregnant, because the elasticity of the muscle fibers in the scar area located in the lower uterus will be significantly reduced, which will lead to weak uterine contractions, resulting in postpartum hemorrhage. At the same time, the scar will also cause certain negative effects on the recovery of the uterus. This leads to endometrial and pelvic infections, which aggravate postpartum morbidity and pain in mothers. Therefore, drugs that can increase uterine contractions should be used to reduce the risk of postpartum hemorrhage [1–3]. Therefore, we showed in this study the effect of carbetocin on intraoperative blood loss and thickness of myometrium during a cesarean section of full-term pregnancy scar uterus.

RETRACTED

## 2. Materials and Methods

Pregnant women with full-term gestational scar uterus who underwent cesarean section from March 1, 2021, to April 30, 2022, were retrospectively collected and divided into a reference group (using oxytocin) or a study group (using carbetocin). Inclusion criteria were as follows: full-term pregnancy; scarred uterus; cesarean section required; and no related treatment was performed prior to inclusion in the study. Exclusion criteria were as follows: coagulation dysfunction; malignant tumors; chronic diseases such as diabetes, pregnancy-induced hypertension, etc.; mental illness; or allergic to drugs.

The clinical data of the two groups were retrospectively collected, and the operation time, intraoperative blood loss, hospital stay, uterine contraction effect, changes in the myometrium, and complications were compared between the two groups. All patients in this study gave informed consent. This study was approved by the institutional ethical committee of our hospital.

All cases underwent cesarean section of the lower uterine segment after spinal anesthesia. The control group was given 100 micrograms of oxytocin, and the study group was given 100 micrograms of carbetocin during c-section.

### 2.1. Statistical Methods

Data were analyzed by SPSS21.0 ((SPSS, Chicago, IL, USA), in which the ^2^ (%) tests were performed for the count data, and the *t*-test (*x* ± *s*) tests were performed for the measurement data. A two-sided*p* < 0.05 was determined as the threshold of statistical significance.

## 3. Results

### 3.1. General Information of the Two Groups of Patients

There was no significant difference in clinical characteristics between the two groups (Table 1).

### 3.2. Comparison of Operative Time, Intraoperative Bleeding, and Hospitalization Time

There were significant differences in operation time (82.18 ± 10.01 vs 104.28 ± 10.33), intraoperative bleeding (210.36 ± 25.89 vs 316.27 ± 20.57), hospital stay (5.86 ± 2.51 vs 7.86 ± 2.57) between the study group and the reference group (*p*=0.0001, 0.005, and 0.006, respectively). See Table 2 for details.

### 3.3. Comparison of Adverse Events

There was a significant difference in the incidence of postoperative adverse events between the study group and the control group (*p*=0.001). See Table 3 for details.

### 3.4. Comparison of Uterine Thickness

There were significant differences in uterine fundus wall thickness (9.18 ± 1.01 vs 7.28 ± 1.33), anterior wall thickness (8.36 ± 1.89 vs 6.27 ± 1.57), and posterior wall thickness (8.86 ± 1.51 vs 6.86 ± 1.57) between the study group and the control group (*p*=0.0004, 0.003, and 0.001, respectively). See Table 4 for details.

RETRACTED

### 3.5. Comparison of Uterine Contraction Effect

There was a significant difference in obvious uterine contraction effect between the study group (53/59) and the reference group (36/44, *p*=0.005, Table 5).

### 3.6. Comparison of Sex Hormone Levels

Before c-section, there were no significant differences in estradiol (E2, (75.03 ± 9.15 vs 74.13 ± 9.07), luteinizing hormone (LH, 3.65 ± 4.51 vs 13.52 ± 4.42), or follicle-stimulating hormone (FSH, 5.52 ± 1.51vs 5.54 ± 1.35) between the study group and the reference group (*p*=0.596, 0.840, and 0.940, respectively). However, after c-section, there were significant differences in E2 (60.96 ± 12.35 vs 66.37 ± 10.07), LH (7.65 ± 2.21 vs 9.25 ± 3.35), FSH (2.08 ± 0.79 vs 3.59 ± 0.51) between the study group and the control group (*p*=0.011, 0.001, and 0.005, respectively, Table 6).

## 4. Discussion

In recent years, due to the continuous development of anesthesia and cesarean section technology, the incidence of cesarean section in China has been as high as 80% in some places. With the implementation of two- and three-child policies, the cicatricial uterus is more common in obstetrics [4]. Evidence shows that when the uterus contracts during the delivery process, the pressure in the uterine cavity will increase, which may cause the rupture of the uterine scar. Furthermore, the elastic plasticity and contractility of the local muscles will be reduced in the scarred uterus, resulting in postpartum hemorrhage. By 6 weeks after a natural delivery, the uterine lining has completely healed, and the whole uterus will return to normal [5–7]. However, this procedure is significantly slowed down in the scarred uterus, and the lochia is difficult to be excreted completely, which affects the contractility of the uterus, prolongs the recovery time of the uterus, and causes poor uterine involution.

Because uterine atony is an important factor leading to massive postpartum hemorrhage, oxytocin-family drugs are used in the routine cesarean section to decrease the risk of postpartum hemorrhage. Oxytocin works quickly, but its half-life is generally 3–4 minutes, requiring multiple or continuous applications. When the dose exceeds 60 U, there will be obvious receptor saturation, which significantly weakens the effect on the lower uterine muscle group. In addition, taking large doses of oxytocin can also cause side effects such as hypotension and arrhythmia. Our study showed that carbetocin has a good hemostatic effect, and the effect is rapid and long-lasting [8–10]. This method has been well applied in the cesarean section of pregnancy with a uterine scar.

RETRACTED

Because fibrous scars significantly reduce the contraction and elongation of the uterus, the scarred uterus is likely to have uterine rupture during pregnancy, vaginal delivery is not recommended. Cesarean section is a common gynecological operation, and its surgical methods and procedures have become mature [11]. But postpartum hemorrhage remains a serious surgical complication that can cause maternal death. In a scarred uterus, the contractile function of the uterine muscle fibers is disrupted, thereby increasing the tension on the surrounding muscle fibers. Therefore, postpartum hemorrhage is common. Improving uterine contractile function is an important measure to prevent postpartum hemorrhage [12, 13]. Oxytocin, misoprostol, ergometrine, etc. are all drugs that can promote uterine contractions. Oxytocin is currently the most often used drug in Obstetrics. It binds to the receptors in the upper uterine segment, and after the receptor site is saturated, it promotes the contraction of the upper uterine segment, but a further increase in the dosage is ineffective anymore. Misoprostol, a derivative of prostaglandins, has a strong effect on smooth muscle contraction, but can also cause side effects such as fever, nausea, and vomiting. Carbetocin is a synthetic, long-acting oxytocin analog with stimulant effects. It can also combine with oxytocin receptors to cause uterine smooth muscle contraction, and hemostasis can be achieved by squeezing blood vessels in the muscle layer [14, 15]. In this study, the operation time, intraoperative bleeding, and hospital stay of the study group were all less than those of the control group. The incidence of postoperative adverse events in the study group was also lower than that in the control group. The uterus in the study group was thicker than that in the control group, and the uterine contraction effect was also more obvious than that in the control group, which further showed the superiority of carbetocin. However, the application of carbetocin in other severe conditions [16–23], as well as its efficacy compared with other choices [24] still needs to be validated.

To sum up, the use of carbetocin in the cesarean section of the full-term scarred uterus has a significant effect, which can effectively shorten the operation time, reduce the amount of intraoperative blood loss, and promote the recovery of the thickness of the anterior and posterior uterine walls and the myometrium, with fewer adverse events.

RETRACTED

## Figures and Tables

**Table 1:** General information of patients.

Generally	Study group	Reference group	*t/χ * ^*2*^	*p*
*n*	59	44		
Age	28.43 ± 4.39	27.51 ± 4.92	1.812	0.074
Parity			10.853	0.791
1	33	25		
>1	26	19		
Nationality			4.927	0.858
Han	56	42		
Other	3	2		
Education level			15.864	0.749
Primary school	11	5		
Junior high school	13	9		
High school	17	11		
University and above	18	19		

**Table 2:** Comparison of bleeding between two groups of patients ($\bar{x}\pm s$).

Group	Operation time (min)	Intraoperative blood loss (ml)	Hospital stay (d)
Reference group (*n* = 44)	104.28 ± 10.33	316.27 ± 20.57	7.86 ± 2.57
Study group (*n* = 59)	82.18 ± 10.01	210.36 ± 25.89	5.86 ± 2.51
*T*	7.943	11.274	9.538
*p*	0.001	0.005	0.006

**Table 3:** Comparison of adverse reactions between the two groups of patients ($\bar{x}\pm s$).

Group	Headache	Dizziness	Nausea	Vomit	Total incidence
Reference group (*n* = 44)	3	4	3	1	11 (25.00)
Study group (*n* = 59)	2	1	2	0	5 (8.47)
*t*					11.139
*p*					0.001

**Table 4:** Comparison of uterine thickness between two groups of patients ($\bar{x}\pm s$).

Group	Bottom wall (mm)	Front wall (mm)	Back wall (mm)
Reference group (*n* = 44)	7.28 ± 1.33	6.27 ± 1.57	6.86 ± 1.57
Study group (*n* = 59)	9.18 ± 1.01	8.36 ± 1.89	8.86 ± 1.51
*T*	10.153	9.365	11.427
*P*	0.004	0.003	0.001

**Table 5:** Comparison of uterine contraction effect between two groups of patients (*n*, %).

Group	Obvious contractions	Subtle contractions
Study group (*n* = 59)	55 (93.22)	4 (6.78)
Reference group (*n* = 44)	35 (79.55)	9 (20.45)
*chi-square test*		4.274
*p*		0.039

**Table 6:** Changes in *T*, LH, and FSH levels before and after birth ($\bar{x}\pm s$).

Group	*n*	E2 (ng/dl)		LH (mIU/ml)		FSH (mIU/ml)	
		Prenatal	Postpartum	Prenatal	Postpartum	Prenatal	Postpartum
Study group	59	75.03 ± 9.15	60.96 ± 12.35a	13.65 ± 4.51	7.65 ± 2.21a	5.52 ± 1.51	2.08 ± 0.79
Reference group	44	74.13 ± 9.07	66.37 ± 10.07a	13.52 ± 4.42	9.25 ± 3.35a	5.54 ± 1.35	3.59 ± 0.51
*t*	—	0.532	12.583	0.202	8.934	0.075	10.033
*p*	—	0.596	0.011	0.840	0.001	0.940	0.005

## Data Availability

The data used to support the findings of this study are available from the corresponding author upon request.
